This article has been retracted.

# Does globalization matter in the relationship between renewable energy consumption and economic growth, evidence from Asian emerging economies

**DOI:** 10.1371/journal.pone.0289720

**Published:** 2023-08-16

**Authors:** Jinjin Zhang, Zixuan Li, Arshad Ali, Jinshu Wang

**Affiliations:** 1 Centre for Public Policy and the Innovation of Social Management, Henan Normal University, Xinxiang, China; 2 School of Business, University of Leeds, Leeds, United Kingdom; 3 Institute of Economics and Management, North East Agricultural University, Harbin, China; 4 Academy of Visual Art, Hong Kong Baptist University, Kowloon, Hong Kong; University of City Island, CYPRUS

## Abstract

The study aims to investigate the impact of social, economic and political globalization on the renewable energy-economic growth nexus in a panel of six Asian emerging economies over the period 1975–2020. The results of the CS-ARDL approach show that renewable energy consumption contributes significantly to long run economic growth. Economic and political globalization firmly hold back economic growth, while social globalization directly promotes economic growth. The nonlinear effects of political, social, and economic globalization on economic growth clearly demonstrate the validity of the inverted U-shaped relationship between political globalization, economic globalization, and economic growth, and the U-shaped relationship between social globalization and economic growth. The study also found that economic, social and political globalization moderated the impact of renewable energy on boosting economic growth. Based on the renewable energy consumption model, it is revealed that economic growth significantly promotes long run renewable energy consumption. Economic, social, and political globalization have significantly boosted long run renewable energy consumption. However, the nonlinear effect model reflects a U-shaped relationship between globalization indicators and renewable energy consumption. The interaction of political, economic, and social globalization with economic growth has also witnessed an increase in renewable energy consumption, which supports the scale effect hypothesis. The causality test concludes that there is a two-way causal relationship between renewable energy consumption and economic growth, thus supporting the feedback hypothesis. The policy implications for Asian emerging economies are discussed based on the empirical analysis of this study.

## 1. Introduction

In recent years, policy circles and academia have paid great attention to issues related to economic growth and renewable energy consumption. Numerous theoretical and empirical studies have been feverishly scrutinizing the interplay between economic growth and various aspects of energy consumption, including the mechanisms by which renewable energy consumption can sustain economic growth in the long run [1–3]. The ongoing debate on the relationship between economic growth and renewable energy consumption has produced conflicting signals and remains inconclusive [4, 5]. For example, few studies show a weak relationship between economic growth and renewable energy consumption. Another stream of empirical research revealed a possible causal relationship between economic growth and renewable energy consumption, leading to the development of four hypotheses: neutral [4, 6–9], feedback [10–12], growth [13, 14], and conservation [15–17] hypotheses. Groundbreaking empirical research focuses on bivariate models to detect causal relationships between renewable energy consumption and economic growth. Recent empirical studies on the link between renewable energy consumption and economic growth employ multivariate and advanced econometric methods to explore the direction of the causal relationship between renewable energy consumption and economic growth. Thus, other variables such as infrastructure development, financial development, institutional quality, capital, energy prices, urbanization, industrialization, carbon emissions, and industrialization have been added to empirical models of the relationship between renewable energy consumption and economic growth to prevent variable omission bias [18–28]. However, there is limited literature on the important role of social, political and economic globalization in the link between renewable energy consumption and economic growth. This raises concerns about the impact of structural and energy efficiency policies in both advanced and developing economies, as the associated policy consequences are temporary.

Globalization is said to facilitate technology transfer, thereby affecting renewable and non-renewable energy use and economic growth [29–31]. Moreover, globalization may stimulate the demand for factors of production to facilitate the production of goods, thereby promoting the use of renewable and non-renewable energy sources and economic growth [32–34]. It has also been suggested that globalization may promote specialization in production, thereby driving economies of scale and higher economic production [35, 36]. To support the recognition of the future impact of globalization on economic growth and renewable energy consumption, it is crucial to strengthen the link between renewable energy consumption and economic growth through social, political and economic indicators of globalization. Studies also use foreign direct investment (FDI) and trade as alternatives to globalization to explore their effects on economic growth or renewable energy consumption [37–39]. However, globalization also has political and social dimensions and is not limited to trade and foreign direct investment, so few empirical studies have revealed the impact of social, political and economic globalization on the link between renewable energy consumption and economic growth, especially in Asian emerging economies. Thus, this study employs panel data techniques to investigate the impact of social, economic, and political globalization on the link between renewable energy consumption and economic growth in China, India, Bangladesh, South Korea, Singapore, and Taiwan during the period 1975 to 2020. The consideration of the above-mentioned countries is because these countries have high energy utilization rate and fast economic growth, and bear the brunt of the globalization process [40, 41]. Thus, consideration of the role of globalization in renewable energy consumption and economic growth in emerging Asian economies can make a significant contribution to the current debate on the impact of globalization on the link between economic growth and renewable energy consumption.

This study contributes to the existing literature on globalization, renewable energy consumption, and economic growth in selected Asian emerging economies by precisely addressing three key questions. Different from the traditional methods used in previous panel studies, this study adopts the CS-ARDL method, which is robust to cross-sectional dependence (CD), heterogeneity and endogeneity, to explore the impact of globalization indicators (social, economic and political) on renewable energy consumption and economic growth. Second, in contrast to previous empirical studies on the subject, this study examines the moderating effects of economic growth and globalization indicators on renewable energy consumption, and the moderating role of renewable energy consumption and globalization indicators on economic growth. Finally, this study explores the non-linear effects of social, political, and economic globalization on renewable energy consumption and economic growth as an extension of the empirical literature.

## 2. Literature review

The literature review in this section focuses on the role of globalization in the link between renewable energy consumption and economic growth. The literature is organized into three core sections: the link between renewable energy consumption and economic growth; the association between globalization and economic growth; and the link between globalization and renewable energy consumption. As noted in each subcategory, findings on these topics are mixed.

### 2.1 The link between renewable energy consumption and economic growth

A large literature reveals the link between renewable energy consumption and economic growth, reporting inconclusive empirical and theoretical evidence. However, research also shows a weak relationship between renewable energy consumption and economic growth [42–44]. Other researchers have identified possible causal relationships between renewable energy consumption and economic growth that fall into four central hypotheses [45, 46]. First, the growth hypothesis proposes that the expansion of renewable energy consumption will lead to the extension of economic growth [47–50]. Second, conservative assumptions suggest that higher economic growth can stimulate renewable energy consumption [16, 51–53]. Studies report evidence for feedback hypothesis based on two-way causality between renewable energy consumption and economic growth [13, 28, 54–56]. The neutral hypothesis suggests an independent link between renewable energy consumption and economic growth [4, 6–9]. Results related to these assumptions fluctuate according to the methodology used, energy dimension, region and income grouping countries.

[57] illustrated that renewable energy consumption made a significant contribution to economic growth; and supported a feedback hypothesis based on a two-way causal relationship between renewable energy consumption and economic growth in the Turkish economy. [58] reveal that a shock to renewable energy consumption leads to a decline in real GDP per capita, while real GDP per capita increases with a shock to nonrenewable energy consumption. [59] investigate the causal relationship between renewable energy consumption and economic growth by conducting a Granger causality test for 12 EU countries over the period 1990–2014. The findings support the feedback hypothesis by suggesting a long-term two-way causal relationship between renewable energy consumption and economic growth. However, in the short term, the results support conservative assumptions based on a one-way causal relationship from economic growth to renewable energy consumption. [60] establishes a dynamic causal relationship between renewable energy prices and economic growth using a Markov switching vector autoregressive (MS-VAR) model in the cases of Canada, New Zealand, and Norway. The results highlight a one-way link from economic growth to renewable energy consumption in Canada and New Zealand, thereby supporting the conservative assumption. [61] employ a bootstrap panel causality test to explore the causal relationship between renewable energy consumption and economic growth over the period 1990–2015 in 15 emerging countries. The analysis provides evidence for the neutral hypothesis for all selected countries. [25] asserts the conservative hypothesis by revealing that there is a one-way causal link from non-renewable energy consumption to economic growth, while the neutral hypothesis is supported based on the absence of a causal relationship between renewable energy consumption and economic growth in PIMC countries. [52] concluded that using a Fourier causality test, the energy-led growth hypothesis is valid for both energy sources in the United States, India, the United Kingdom, and Spain, while the non-renewable energy-led growth hypothesis is valid for Italy. The conservation hypothesis applies to energy in Germany and renewable energy in China.

Evidence for the direction of causality between renewable energy consumption and economic growth is also mixed for individual countries. [62] use a VECM model to reveal short- and long-term causal relationships between renewable energy consumption and economic growth in Saudi Arabia over the period 1990–2020. The results support the feedback hypothesis, as there is a short- and long-term bidirectional causal relationship between renewable energy consumption and economic growth. [63] examines the direct and indirect effects of renewable energy on economic growth in Ghana over the period 1990–2015 using Granger causality tests and a mediation model. The results identify the feedback hypothesis between renewable energy consumption and economic growth. [64] adopted the causality test of Toda and Yamamoto (1995) and showed no significant causal relationship between renewable energy consumption and economic growth in Morocco, thus supporting the neutral hypothesis. [65] adopted a Granger causality test for the period 1990–2019, revealing a two-way causal relationship between renewable energy consumption and economic growth, supporting the feedback hypothesis in Argentina.

### 2.2 The relationship between globalization and economic growth

Globalization includes economic, political and social dimensions and is not limited to trade openness. As this phenomenon of globalization affects the development of a country is still a controversial topic because its impact varies according to the dimensions and relative resources of the country [66]. The role of globalization in development defines conflicting perspectives advanced by theoretical and empirical growth research. Globalization is said to drive economic growth [67, 68], through technological diffusion, effective resource allocation, capital augmentation and improved factor productivity [69–71]. Globalization leads to the transfer of advanced technology from developed to developing countries, thereby promoting the division of labor to benefit more from a country’s comparative advantage in producing different specialized activities [72, 73]. [74] pointed out that overall globalization has a positive impact on economic growth, while the impact of fragmented globalization on economic growth shows that the social and political levels promote economic growth, while the economic level destroys economic growth in low-income countries. [75] use the Pooled Autoregressive Distribution Lag (ARDL) method to conclude that globalization has a positive effect on economic growth, which may not be sustained by rising interest rates and inflationary pressures, however, economic globalization can be used as a tool to stimulate investment, curbing corruption and subsequently sustaining economic growth in South Asian economies.

Conversely, globalization can undermine growth in countries with weak institutions and political instability [30, 76]. Few researchers argue that the impact of trade on economic growth is limited by a country’s structural progress and claim no strong positive effects [77, 78]. Other research has shown that lack of consideration of important growth indicators reduces the positive impact of globalization on growth by linking such evidence to globalization indices [79, 80]. According to the Stolper-Samuelson Heckscher-Ohlin theorem, countries with relatively scarce resources will lose from freer trade, while countries with relatively abundant resources will benefit [81]. Thus, people worry about the distributional effects of globalization on the economy, while classical and neoclassical literature affirms the benefits of globalization. [82] contended that when globalization affects labor markets with gender consequences, the distributional effects of traded inputs, non-traded goods and outsourcing may affect social justice. For instance, when low-income countries have a comparative advantage in producing low-skilled labour-intensive goods, low-skilled women enter the labor force.

Trade liberalization is good for economic growth, which is concluded after reviewing the historical evidence on the link between globalization and economic growth [83], however, successful capital liberalization requires high-quality systems [84, 85]. [86] demonstrated that Globalization influence institutional significantly, such institutional reforms in turn facilitate economic growth in East Asian countries. Using the KOF globalization index and institutional governance indicators, [87] adopts a two-step systematic GMM approach to a sample of 45 Asian economies and reveals their impact on GDP growth during 2003–2017. The results show that globalization makes a significant contribution to economic growth through sound regulatory controls and political stability.

### 2.3 The relationship between globalization and renewable energy consumption

[88] investigate the role of economic globalization on renewable energy consumption in panel data covering 30 OECD countries from 1970 to 2015. The results show that higher levels of economic globalization promote the development of renewable energy, and the evidence for different measures of economic globalization is strong. However, [89] uses panel quantile regression for OECD countries to determine that economic globalization reduces renewable energy consumption, while overall globalization (economic, social, and political) increases renewable energy consumption. Similarly, [90] conclude that the short- and long-term overall globalization process and its long-term economic and political globalization dimensions have a significant positive impact on Turkey’s renewable energy consumption. However, social globalization does not have any significant impact on Turkey’s short- and long-term renewable energy consumption. [91] uses a nonlinear PSTR model to reveal the link between globalization, renewable energy consumption, and carbon emissions for 33 OECD countries during the period 2000–2018. The results show that with the increase of the level of globalization, the carbon emission reduction effect of renewable energy is stimulated, that is, globalization changes the relationship between renewable energy consumption and carbon emissions in OECD countries.

In conclusion, views vary on the link between renewable energy consumption and economic growth; the association between globalization and economic growth; and the relationship between globalization and renewable energy consumption. However, no studies have considered globalization as a channel influencing the link between renewable energy consumption and economic growth. For the most part, these relationships are explored independently in each model; thus, further research on the role of globalization in creating a win-win situation for specific emerging Asian economies is urgently needed.

## 3. Model specification, variable data measurements, and sources and methods

This study reveals the impact of disaggregated globalization (social, political, and economic globalization) on renewable energy consumption and economic growth in emerging Asian economies. To detect this relationship, two main empirical models were developed.

### 3.1 Economic growth model

Following [92–95], the Cobb-Douglas production function is extended to explore the impact of renewable energy consumption and globalization on economic growth. [92] enhanced the Cobb-Douglas production function by including renewable energy consumption and non-renewable energy consumption, revealing the impact of renewable energy use, non-renewable energy use, capital and labor on economic growth. [93] used financial globalization and other labor and capital control factors in the model to reveal its impact on economic growth. Thus, the model can be more fully interpreted as economic growth (Y) as a function of capital (K), labor (L), renewable energy consumption (RE), disaggregated globalization (GLO), and other variables (Z) that may affect economic growth with potential.


Y=f(K,L,RE,GLO,Z) (1)

The above function can be expressed in log-linear form as:

$$\ln Y_{i,t}=\alpha_{0}+\alpha_{1}\ln K_{i,t}+\alpha_{2}\ln L_{i,t}+\alpha_{3}\ln RE_{i,t}+\alpha_{4}\ln GLO_{i,t}+\alpha_{j}\ln Z_{i,t}+\mu_{i,t}$$ (2)

Few studies have emphasized that the impact of globalization on economic growth is not always linear but nonlinear [96–98]. The above equation based on this argument can be augmented with a quadratic term for globalization to capture its non-linear effects:

$$\ln Y_{i,t}=\alpha_{0}+\alpha_{1}\ln K_{i,t}+\alpha_{2}\ln L_{i,t}+\alpha_{3}\ln RE_{i,t}+\alpha_{4}\ln GLO_{i,t}+\alpha_{5}\ln GLO_{i,t}^{2}+\alpha_{j}\ln Z_{i,t}+\mu_{i,t}$$ (3)

Uncovering the moderating role of decentralized globalization in the link between renewable energy consumption and economic growth, Eq (3) is further extended to include an interaction term (GLO × RE). Inserting an interaction term into this model is crucial as it may help to understand how globalization is intertwined with the impact of renewable energy consumption on economic growth:

$$\ln Y_{i,t}=\alpha_{0}+\alpha_{1}\ln K_{i,t}+\alpha_{2}\ln L_{i,t}+\alpha_{3}\ln RE_{i,t}+\alpha_{4}\ln GLO_{i,t}+\alpha_{5}\ln{\left(GLO*RE\right)}_{i,t}+\alpha_{j}\ln Z_{i,t}+\mu_{i,t}$$ (4)

Where *α*_0_, *α*_1_, *α*_2_,….. *α*_*j*_ reflect parameters to be estimated and *μ*_*i*,*t*_ is the random error term in the economic growth model.

### 3.2 Renewable energy consumption model

Following [99–101], the renewable energy consumption model can be specified as economic growth (Y), labor force (L), capital (K), decomposed globalization (GLO) and other variables (Z), which impact on renewable energy consumption.


RE=f(Y,K,L,GLO,Z) (5)

Renewable energy consumption model in the log linear form can be specified as:

$$\ln RE_{i,t}=\beta_{0}+\beta_{1}\ln K_{i,t}+\beta_{2}\ln L_{i,t}+\beta_{3}\ln Y_{i,t}+\beta_{4}\ln GLO_{i,t}+\beta_{j}\ln Z_{i,t}+\varepsilon_{it}$$ (6)

Eq (6) can be augmented with a quadratic term for globalization to capture its non-linear effects:

$$\ln RE_{i,t}=\beta_{0}+\beta_{1}\ln K_{i,t}+\beta_{2}\ln L_{i,t}+\beta_{3}\ln Y_{i,t}+\beta_{4}\ln GLO_{i,t}+\beta_{5}\ln GLO_{i,t}^{2}+\beta_{j}\ln Z_{i,t}+\varepsilon_{i,t}$$ (7)

Uncovering the moderating role of decentralized globalization in the link between economic growth and renewable energy consumption, Eq (7) is further extended to include an interaction term (GLO × Y).


$$\ln RE_{i,t}=\beta_{0}+\beta_{1}\ln K_{i,t}+\beta_{2}\ln L_{i,t}+\beta_{3}\ln Y_{i,t}+\beta_{4}\ln GLO_{i,t}+\beta_{5}\ln{\left(GLO*Y\right)}_{i,t}+\beta_{j}\ln Z_{i,t}+\varepsilon_{i,t}$$ (8)

Where *β*_0_, *β*_1_,*β*_2_,….. *β*_*j*_ reflect parameters to be estimated and *ε*_*i*,*t*_ is the random error term in the renewable energy consumption model.

### 3.3 Variable data descriptions, measurements and sources

The Table 1 below highlights variable measurements and descriptions and data sources, renewable energy consumption data measured in million tons of oil equivalent (Mtoe), obtained from the [102]. Subdivided globalization includes economic globalization, social globalization and political globalization. The data of economic globalization can be obtained by making an index of the indicators of trade globalization and financial globalization. Similarly, social globalization can also be measured by making an index on the indicators of personal globalization, information globalization and cultural globalization. However, political globalization data can directly be obtained from [103]. Likewise, data for the Social Globalization Index and the Economic Globalization Index are also available from the [103]. GDP can be used as a proxy for economic growth, and data on GDP and capital in constant 2015 US$ are available from WDI [104]. Employed labor force data in millions is also available from WDI [104].

**Table 1:** Description and measurement of variables and data sources.

Variables	Description	Measurment	Sources
GDP	Gross Domestic Product	Constant 2015 US$	WDI, World Bank (2022)
EGLO	Economic globalization	Economic globalization index	KOF Swiss Economic institute (2022)
REC	Renewable Energy Consumption	Million tons of oil equivalent (Mtoe)	OECD (2020)
SGLO	Social globalization	Social globalization index	KOF Swiss Economic institute (2022)
PGLO	Political globalization	Percentage	KOF Swiss Economic institute (2022)
K	Gross fixed capital formation	Constant 2015 US$	WDI, World Bank (2022)
L	Employed labor force	Million	WDI, World Bank (2022)

### 3.4 Cross-sectional dependence and slope heterogeneity tests

As interdependence increases, panels may have significant cross-sectional dependence (CSD), so more stringent tests are needed to examine for cross-sectional dependence across countries. Thus, the current study explicitly examines cross-sectional correlation tests to address issues with panel data estimation and to ensure that empirical estimates are unbiased, consistent, and valid. Primarily Pesaran CSD, Pesaran scaled LM, bias-corrected scaled LM and Breush-Pegan LM test introduced by [105–108], expressed by the following Eqs (9&10), respectively.

$$CSD=\sqrt{\frac{2T}{N(N-1)}}(\sum_{i=1}^{N-1}\sum_{K=i+1}^{N}\hat{\beta }ik)∼N(0,1)\;I,k$$ (9)

CSD=(1,2,3,…..45,…….N)

$$M=\sqrt{\frac{2T}{N(N-1)}}(\sum_{i=1}^{N-1}\sum_{K=i+1}^{N}\hat{\beta }\;ik)\left[\frac{(T-K){\hat{\beta }}_{ik}^{2}-(T-K){\hat{\beta }}_{ik}^{2}}{Var(T-K){\hat{\beta }}_{ik}^{2}}\right]$$ (10)

where the symbols T and N replicate the sample size (period) and panel size (cross-section), respectively. It turns out that panel datasets with cross-sectional dependencies will be more prominently used in second-generation panel data techniques. More appropriate steady-state results can be established using second-generation panel stationary testing.

### 3.5 Panel unit root tests

First-generation panel stationary tests, Augmented Dickey Fuller; Phillip Perron; Lin and Chu; Levin; Hadri; Breitung; Im, Pesaran, and Shin failed to account for cross-sectional dependencies in longitudinal datasets. Thus, to reduce this concern, the current study used second-generation panel unit root tests, namely the cross-sectional Im, Pesaran and Shin (CIPS) test developed by [109], and the cross-sectional augmented Dickey-Fuller (CADF) test. These panel unit root tests are more robust and perform better due to the asymptotic assumption and not requiring (N⁓∞). CADF and CIPS panel unit root tests can be used to generate accurate information about the order of integration of the series. Eq (11) below represents the CADF panel unit root test.


$$\Delta z_{\mathrm{it}}=\alpha_{i}+\beta_{i}z_{\mathrm{it}-1}+\kappa_{i}{\bar{z}}_{t-1}+\Psi \Delta {\bar{z}}_{t}+\mu_{it}$$ (11)

Substituting the lag term (t-1) in Eq (11) yields the following Eq (12)

$$\Delta z_{\mathrm{it}}=\alpha_{i}+\beta_{i}z_{\mathrm{it}-1}+\kappa_{i}{\bar{z}}_{t-1}+\sum_{j=0}^{k}\Psi_{ij}\;\Delta {\bar{z}}_{it-1}+\sum_{j=0}^{k}\lambda_{ij}\;\Delta z_{it-1}\upsilon_{\mathrm{it}}$$ (12)

where ${\bar{z}}_{it-1}$ and Δ*z*_*it*−1_ signify the lag level of each cross section and the mean value of the first-order difference operator, respectively. Eq (13) below represents the second-generation CIPS unit root test.


$$CIPS=N^{-1}\sum_{i=1}^{N}\lambda_{i}(N,T)$$ (13)

The coefficient *λ*_*i*_ (*N*, *T*) the test statistic of CADF, so replacing *λ*_*i*_ (*N*, *T*) with CADF, the following Eq (14) can be obtained.


$$CIPS=N^{-1}\sum_{i=1}^{N}\lambda_{i}CADF$$ (14)

### 3.6 Panel cointegration test

The results of the unit root approach describe integration at mixed levels, such as I(0) and I(1), so we turned to cointegration analysis, using the [110] test to estimate possible cointegration relationships in panel data. This approach is consistent even in the presence of cross-sectional dependencies, heterogeneity, and non-stationary regressors, and relies heavily on Durbin Hausman’s principles to generate two statistics. Long-term relationships under heterogeneity can be revealed with the first statistic (DHg), while relationships under the assumption of panel data homogeneity can be explored with the second statistic (DHp). The explanation of the Durbin-Hausman test statistic is determined as:

$$DH_{g}=\sum_{i=1}^{n}{\hat{s}}_{i}({\overset{ˇ}{\emptyset }}_{i}+{\hat{\emptyset }}_{i}{)}^{2}\sum_{t=2}^{Т}{\hat{e}}_{it-1}^{2}$$ (15)

$$DH_{p}={\hat{s}}_{i}({\overset{ˇ}{\emptyset }}_{i}+{\hat{\emptyset }}_{i}{)}^{2}\sum_{i=1}^{n}\sum_{Т=2}^{Т}{\hat{e}}_{it-1}^{2}$$ (16)

The null hypothesis of the Durbin Hausman panel statistic (DHp) can be expressed as H_0_: ∅_*i*_ = 1 for all i, where, i = 1,2,…..n. However, the alternative hypothesis can be exposed as $H_{i}^{P}:\emptyset_{i}=\emptyset_{i},\emptyset_{i}$ < 1for all i. In contrast, the null hypothesis of the Durbin Hausman group statistic (DHg) can be shown as H_0_: ∅_*i*_ = 1 for all i, against the alternative hypothesis as $H_{i}^{g}:\emptyset_{i}=\emptyset_{i},\emptyset_{i}$ < 1for all i.

### 3.7 Long run estimates

The next step after cointegration analysis is to estimate the long-term relationships among the proposed variables in the model. This study uses the CS-ARDL approach proposed by [111], which has recently outperformed traditional estimation techniques (i.e., OLS, FMOLS, DOLS) in estimating short- and long-run elasticities. The CS-ARDL estimation technique can account for cross-sectional dependence, serial correlation, endogeneity, and heterogeneity issues [112].

The CS-ARDL equation can be expressed as:

$$\Delta {\mathrm{EF}}_{\mathrm{i,t}}=\emptyset_{i}+\sum_{j=1}^{p}\emptyset_{it}\Delta {\mathrm{EF}}_{\mathrm{i,t}}‐j+\sum_{j=0}^{p}{\overset{´}{\emptyset }}_{it}{\mathrm{AEV}}_{\mathrm{i,t}}‐j+\sum_{j=0}^{p}{\overset{´}{\emptyset }}_{it}{\bar{Z}}_{t}‐j+\mu_{\mathrm{i,t}}$$ (17)

The cross-sectional average can be expressed as

${\bar{Z}}_{t}$ ($\Delta {\bar{EF}}_{t},{\bar{AEV}}_{t}$), Z represents the set of explanatory variables. The Augmented Means Group (AMG) estimator developed by [113] is also used in this study as a complement to the CS-ARDL approach. This method can overcome the problems of cross-sectional dependence, slope heterogeneity and endogeneity of panel data and provide long-term results, so the AMG strategy can be used as a robustness test.

### 3.8 Granger causality test

The Granger causality test of [114] can be used after long-term estimated parameters to reveal bidirectional causality between variables of interest. This method is not subject to any restriction of T>N, and is very flexible and applicable. This test is suitable for heterogeneous and unbalanced panels. This method provides robust conclusions even for small samples and cross-sectional dependence, as recognized by Monte Carlo simulations [115]. The Dumitrescu-Hurlin causality test equation can be expressed as:

$$y_{i,t}=\emptyset_{i}+\sum_{j=1}^{p}\partial_{i}^{j}y_{i,t-j}+\sum_{j=1}^{p}\lambda_{i}^{j}z_{i,t-j}$$ (18)

## 4. Analysis results and interpretation

First, cross-sectional dependencies in panel datasets can be detected to obtain robust estimation results. Pesaran Scaled LM, Pesaran CSD, Bias-corrected scaled LM, and BreuschPagan LM tests yielded strong evidence of cross-sectional dependence in the panel datasets for the six emerging Asian countries highlighted in Table 2. Thus, the results obviously illustrate a strong correlation among specific countries in the panel. With the emergence of cross-sectional dependencies in panel datasets, second-generation techniques will produce reliable, robust, efficient, and consistent results.

**Table 2:** Results of cross-sectional dependence tests.

	Breusch-Pagan LM		Pesaran Scaled LM		Biased-corrected Scaled LM		Pesaran CSD	
Variables	Statistics	Probability	Statistics	Probability	Statistics	Probability	Statistics	Probability
lnGDP	351.92***	0.005	38.82***	0.000	54.96***	0.001	32.78**	0.034
lnRE	421.94***	0.007	98.39***	0.000	68.94***	0.000	25.48***	0.009
lnSGLO	269.47***	0.001	87.49***	0.000	37.49***	0.002	37.78***	0.000
lnEGLO	522.98***	0.000	72.83***	0.005	46.84***	0.000	35.28***	0.008
lnPGLO	528.43**	0.031	26.39**	0.039	37.38***	0.000	42.35***	0.000
lnK	684.39***	0.001	91.27***	0.000	43.47***	0.000	36.27***	0.000
lnL	387.21**	0.034	37.21***	0.008	63.32***	0.003	43.29***	0.003

Note: *, **, *** indicate statistical significance levels of 10%, 5%, and 1%, respectively.

The slope heterogeneity results in Table 3 clearly demonstrate heterogeneity problems in the leading models of renewable energy and economic growth, reflecting biases in the results of traditional cointegration techniques and unit root tests. The test statistics of both models are statistically significant, thus, in this case, the most appropriate method adopted in this study is the second-generation unit root test of CADF and CIPS, and the results are summarized in Table 4. The results of the CADF and CIPS tests identify stationary outcomes at 1(1) for the entire variable in the model, allowing cointegration analysis to be used.

**Table 3:** Pesaran and Yamagata slope heterogeneity test results.

Models	Test	Value	Probability
Model-Y	$\overset{ˇ}{\Delta }$	52.37***	0.002
	${\tilde{\Delta }}_{adjusted}$	41.26***	0.003
Model-RE	$\overset{ˇ}{\Delta }$	47.16***	0.005
	${\tilde{\Delta }}_{adjusted}$	65.64***	0.000

Note: *** indicate statistical significance levels of 1%.

**Table 4:** Panel unit root tests.

	CADF		CIPS	
Variables	Level	First difference	Level	Difference
lnGDP	-1.74	-1.02***	-1.81	-3.79***
lnRE	-1.48	-3.37***	-1.58	-2.89***
lnSGLO	-1.84	-3.71***	-1.92	-3.08***
lnEGLO	-1.79	-4.95***	-2.94	-3.68***
lnPGLO	-1.94	-3.85***	-2.26	-4.04***
lnK	-1.69	-2.76***	-1.47	-2.61***
lnL	-1.32	-2.37***	-1.28	-3.21***

**Note:** *, **, *** indicate statistical significance levels of 10%, 5%, and 1%, respectively.

The variable descriptive statistics highlighted in Table 5 reflect an average GDP of $2,096.87 billion for the six largest emerging economies in Asia, showing a large standard deviation for the period 1975–2020. The average levels of social globalization, economic globalization and political globalization are 56.47%, 51.43% and 48.19% respectively, and the deviations are 15.91%, 7.68% and 8.65% respectively. These statistics reflect the greater economic, social and political integration of particular emerging economies with the global economy. The average renewable energy consumption in selected emerging economies in Asia was 6.26 metric tonnes of oil equivalent (Mtoe), with a variation of 0.96 Mtoe. The skewness statistics are positive, reflecting that all variable data are positively skewed. In addition, average gross fixed capital formation (K) and employed labor force (L) recorded $4.89 trillion and 628 million, respectively. The kurtosis results reflect the elongation and peaking phenomenon of capital and GDP data due to large statistics. Also, the Jarque-Bera test reflects the normal distribution of the data for the entire variable, since none of the variables are significant.

**Table 5:** Panel descriptive statistics.

Variables	Average	SD	Max	Min	Kurtosis	Skewness	Jarqua-Bera	Probability
lnGDP	2096.87	838.97	2291.26	654.82	1.74	0.84	1.55	0.43
lnSGLO	56.47	15.91	67.28	36.73	1.46	0.62	1.59	0.13
lnEGLO	51.43	7.68	61.47	47.37	1.58	0.58	1.47	0.29
lnPGLO	48.19	8.65	57.15	43.38	1.69	0.37	1.64	0.38
lnREC	6.26	0.96	9.1397	2.535	1.81	0.48	1.42	0.21
lnK	4.89	0.532	5.63	0.22	1.62	0.78	1.53	0.42
lnL	628.00	86.00	826.00	538.00	1.72	0.64	1.63	0.16

Correlation coefficients and variance inflation factors (VIF) for each variable in Table 6, used to check for multicollinearity problems in the series. The results of the correlation matrix illustrate that social globalization, political globalization, capital and labor force are positively correlated with GDP, while economic globalization, and renewable energy consumption are adversely associated with GDP. The results for the variance inflation factor (VIF) reflect the absence of multicollinearity in the model, as all VIF values are below 5.

**Table 6:** Correlation matrix and VIF tests.

lnGDP		lnSGLO	LnEGLO	lnPGLO	lnREC	lnK	lnL	VIF
lnGDP	1							
lnSGLO	0.858	1						3.48
lnEGLO	-0.975	0.907	1					4.14
lnPGLO	0.418	-0.748	0.839	1				3.08
lnREC	-0.326	-0.357	0.426	0.389	1			3.39
lnK	0.433	0.398	0.305	0.353	0.365	1		3.17
lnL	0.366	0.481	0.526	0.436	0.438	0.435	1	3.28

Next, the [110] cointegration test, which is widely used in the energy growth, globalization-renewable energy consumption, and globalization-economic growth literatures, is applied based on the use of partial integral regressors. This test gives way to accommodating elite characteristics of stationary regressors in the model. The possibility to place partially stationary regressors in the model is a distinguishing feature of the test. Thus, it is more appropriate to use this test in the current study. The results of the Westerlund test highlighted in Table 7 demonstrate the acceptability of the alternative hypothesis, showing cointegration in the panel data for selected emerging Asian economies.

**Table 7:** Westerlund long term cointegration test.

Westerlund (2008) cointegration test	Statistics	P-value
Gt	-8.96***	0.00
Ga	-6.87***	0.00
Pt	9.06***	0.00
Pa	-23.72***	0.00

**Note:** *** indicate statistical significance levels of 1%.

### 4.1 Long-term coefficient estimation of economic growth model

Table 8 highlights the estimated long-run coefficient elasticities of the economic growth model revealed by the CS-ARDL approach. Every 1% increase in renewable energy consumption can significantly boost economic growth by 0.609%. The analysis results show that renewable energy consumption has a significant progressive effect on economic growth. This result identifies renewable energy consumption as a major factor affecting economic growth in selected Asian emerging economies, which is inconsistent with the arguments of classical economics. Thus, implementing policies to expand renewable energy efficiency will boost economic growth in Asian emerging economies, consistent with previous studies by [25, 28, 47, 49, 50, 116–119]. Also, gross fixed capital formation has significantly boosted economic growth in specific emerging Asian economies. Every 1% increase in gross fixed capital formation can significantly promote economic growth by 0.476%. This result is consistent with the neoclassical growth model, which is based on the fact that higher capital accumulation can boost economic growth. Likewise, the employed labor force has a significant positive effect on economic growth in specific emerging Asian economies. Every 1% increase in the employed labor force can significantly boost economic growth by 0.309%.

**Table 8:** Long-term results of CS-ARDL test.

Variables	Coefficients	Standard error	Z-value	P-value
lnGDP = f(InRE, InSGLO, InEGLO, InPGLO, lnK, lnL)				
lnRE	0.609***	0.079	3.204	(0.000)
lnSGLO	0.423***	0.031	4.212	(0.000)
lnEGLO	-0.218***	0.027	-3.074	(-0.003)
lnPGLO	-0.533***	0.058	-5.781	(-0.004)
lnK	0.476***	0.091	4.081	(0.003)
lnL	0.309***	0.042	3.065	(0.003)
ECM(-1)	-0.788***	0.081	-34.782	(0.000)
InGDP = f(InRE, InSGLO, lnEGLO, InPGLO, lnSGLO^2^, lnEGLO^2^, lnPGLO^2^, lnK, lnL)				
lnRE	0.792***	0.091	4.016	(0.002)
lnSGLO	-0.491**	0.017	-2.092	(-0.041)
lnEGLO	0.287***	0.035	4.065	(0.000)
lnPGLO	0.586***	0.042	5.142	(0.004)
lnSGLO^2^	0.307***	0.081	4.215	(0.000)
lnEGLO^2^	-0.176**	0.062	-3.298	(0.027)
lnPGLO^2^	-0.315***	0.071	-4.214	(0.000)
lnK	0.276*	0.037	5.321	(0.063)
lnL	0.327***	0.083	3.257	(0.003)
ECM(-1)	-0.806***	0.0817	-27.078	(0.000)
InGDP = f(InRE, InSGLO, lnEGLO, InPGLO, lnSGLO*lnRE, lnEGLO*lnRE, lnPGLO*lnRE, lnK, lnL)				
lnRE	0.642***	0.082	4.676	(0.003)
lnSGLO	0.391**	0.047	2.082	(0.041)
lnEGLO	-0.297***	0.055	-4.475	(0.000)
lnPGLO	-0.406***	0.042	-5.572	(-0.004)
lnSGLO*RE	0.267***	0.054	3.182	(0.007)
lnEGLO*RE	0.296**	0.015	5.021	(0.038)
lnPGLO*RE	0.326***	0.073	4.324	(0.000)
lnK	0.264**	0.081	2.279	(0.025)
lnL	0.316***	0.043	4.145	(0.000)
ECM(-1)	-0.912***	0.0827	-37.088	(0.000)

**Note:** ***, ** and * indicate statistical significance at 1% level, 5% level and 10% level respectively, where inside in the parentheses are probability values.

Focusing on decomposed globalization, it can be seen from the direct effect model that both political globalization and economic globalization have hindered the economic growth of emerging economies in Asia. For every 1 percentage point increase in political globalization and economic globalization, the economic growth rate can be significantly reduced by 0.218 percentage points and 0.533 percentage points respectively. Hence, economic globalization, including the flow of goods, services, and financial assets, has hindered economic growth in specific emerging Asian economies. This may be because it stimulates expertise in economic sectors with strong comparative barriers to technological innovation, learning by doing, and possible productivity growth that have mostly disappeared in emerging Asian economies [120, 121]. In addition, economic globalization may hinder economic growth through the failure and unemployment of new industries and widening income inequality [122, 123]. Moreover, the negative impact of economic globalization on economic growth is caused by weak institutions in emerging economies, which is consistent with [70, 124, 125]. This result is consistent with [70, 74, 126], also contradicting [75, 127, 128]. Moreover, weak institutions and governance replicate the deterrent effect of political globalization on economic growth in emerging Asian economies. Institutional weaknesses in emerging Asian economies impede growth by undermining the effectiveness of domestic institutions. In view of the restrictive effect of economic and political globalization on the economic growth of Asian emerging economies, political factors reflect economic factors, and the two complement each other. The restrictive effect of political globalization on economic growth is very consistent with the research results of [30, 70, 76, 129, 130]. Conversely, social globalization has accelerated economic growth in Asia’s emerging countries. Thus, given the free flow of communication and information enabled by social globalization through television, telephone, and the Internet, it may stimulate economic growth by lowering transaction costs [66, 131]. This result is consistent with studies by [70, 127, 132].

The non-linear impact of political, economic and social globalization on economic growth shows that political and economic globalization significantly promotes economic growth, while social globalization significantly reduces economic growth. However, the square of political and economic globalization significantly reduces economic growth, while the square of social globalization significantly boosts economic growth in emerging Asian economies. This result clearly proves the validity of the inverted U-shaped relationship between political globalization, economic globalization and economic growth, and the legitimacy of the U-shaped relationship between social globalization and economic growth. This means that economic growth in the short run is boosted by political and economic globalization and held back by social globalization. However, in the long run, economic growth will only increase due to social globalization and decrease due to political and economic globalization. Furthermore, the moderating role of renewable energy in the link between globalization indicators and economic growth suggests that renewable energy consumption interacts with economic, social, and political globalization to promote economic growth in emerging Asian economies.

To check the robustness of the long-term results of the economic growth model through the CS-ARDL test, the AMG estimator is used. Table 9 highlights the AMG estimation results, reflecting broad agreement with the CS-ARDL results in terms of coefficient signs.

**Table 9:** Long-term AMG estimation results for robustness checks.

Variables	Coefficients	Standard error	Z-value	P-value
lnGDP = f(InRE, InSGLO, InEGLO, InPGLO, lnK, lnL)				
lnRE	0.487***	0.059	3.084	(0.002)
lnSGLO	0.203***	0.011	4.952	(0.007)
lnEGLO	-0.178***	0.067	-3.844	(-0.001)
lnPGLO	-0.533***	0.018	5.721	(0.000)
lnK	0.476***	0.051	4.811	(0.005)
lnL	0.309***	0.062	3.745	(0.001)
Constant	-3.788***	0.041	-4.032	(0.009)
Wald	91.263***			
RMSE (sigma)	0.067			
InGDP = f(InRE, InSGLO, lnEGLO, InPGLO, lnSGLO^2^, lnEGLO^2^, lnPGLO^2^, lnK, lnL)				
lnRE	0.402***	0.061	3.436	(0.005)
lnSGLO	-0.571**	0.047	-3.482	(-0.031)
lnEGLO	0.357**	0.065	3.285	(0.033)
lnPGLO	0.476***	0.072	4.262	(0.008)
lnSGLO^2^	0.467***	0.051	5.425	(0.000)
lnEGLO^2^	-0.256***	0.042	-2.438	(0.001)
lnPGLO^2^	-0.465***	0.081	-5.484	(0.000)
lnK	0.356***	0.067	4.561	(0.003)
lnL	0.477***	0.063	4.587	(0.000)
Constant	-0.946***	0.087	-2.938	(0.004)
Wald	83.314***			
RMSE (sigma)	0.042			
InGDP = f(InRE, InSGLO, lnEGLO, InPGLO, lnSGLO*lnRE, lnEGLO*lnRE, lnPGLO*lnRE, lnK, lnL)				
lnRE	0.352***	0.094	4.603	(0.005)
lnSGLO	0.481***	0.041	2.047	(0.001)
lnEGLO	-0.167***	0.059	-4.436	(0.000)
lnPGLO	-0.386***	0.049	-5.547	(-0.009)
lnSGLO*RE	-0.367***	0.051	-3.136	(-0.001)
lnEGLO*RE	-0.516***	0.012	-5.047	(-0.038)
lnPGLO*RE	-0.306**	0.078	-4.358	(-0.000)
lnK	0.394**	0.087	2.218	(0.006)
lnL	0.426***	0.048	4.179	(0.008)
Constant	-0.372***	0.088	-3.63	(0.006)
Wald	89.82***			
RMSE (sigma)	0.064			

**Note:** ***, ** and * indicate statistical significance at 1% level, 5% level and 10% level respectively, where inside in the parentheses are probability values.

Table 10 highlights estimates of renewable energy consumption, showing that economic growth has significantly boosted renewable energy consumption. This clearly shows that demand for renewable energy consumption has been stimulated in Asia’s emerging economies as economic growth picks up. This is because converting raw materials into finished products requires economic agents to use renewable energy through higher economic growth in emerging Asian economies [133, 134]. The result of higher economic growth leading to higher renewable energy consumption is consistent with [15, 135]. The findings also show that capital accumulation significantly increases renewable energy consumption, and argue that capital accumulation and renewable energy are complementary, that is, higher capital stocks in Asian emerging economies will lead to higher renewable energy consumption. In addition, employed labor has a significant adverse effect on renewable energy consumption, suggesting that labor and renewable energy are substitutes, and that an increase in the labor force reduces renewable energy consumption in emerging Asian economies.

**Table 10:** Long-term results of CS-ARDL test.

Variables	Coefficients	Standard error	Z-value	P-value
lnRE = f(InGDP, InSGLO, InEGLO, InPGLO, lnK, lnL)				
lnGDP	0.207***	0.087	3.0261	(0.000)
lnSGLO	0.383***	0.081	4.512	((0.000)
lnEGLO	0.488***	0.067	5.954	(0.005)
lnPGLO	0.373***	0.078	3.371	(0.000)
lnK	0.144***	0.049	3.051	(0.009)
lnL	-0.369***	0.032	4.095	(-0.003)
ECM(-1)	-0.538***	0.099	-23.962	(-0.009)
InRE = f(InGDP, InSGLO, lnEGLO, InPGLO, lnSGLO^2^, lnEGLO^2^, lnPGLO^2^, lnK, lnL)				
lnGDP	0.312***	0.053	3.736	(0.009)
lnSGLO	-0.721***	0.037	-2.312	(-0.001)
lnEGLO	-0.367***	0.055	-2.265	(-0.004)
lnPGLO	-0.406***	0.064	3.422	(-0.007)
lnSGLO^2^	0.467***	0.041	2.075	(0.000)
lnEGLO^2^	0.356**	0.072	3.158	(0.007)
lnPGLO^2^	0.545***	0.091	2.084	(0.000)
lnK	0.416*	0.067	3.301	(0.043)
lnL	-0.267***	0.083	-3.477	(-0.000)
ECM(-1)	-0.916***	0.077	-47.378	(0.000)
InRE = f(InGDP, InSGLO, lnEGLO, InPGLO, lnSGLO*lnGDP, lnEGLO*lnGDP, lnPGLO*lnGDP, lnK, lnL)				
lnGDP	0.292**	0.062	3.096	(0.023)
lnSGLO	0.321***	0.047	2.082	(0.001)
lnEGLO	0.497***	0.035	2.195	(0.000)
lnPGLO	0.196***	0.062	4.012	(0.009)
lnSGLO*GDP	0.487**	0.074	5.052	(0.033)
lnEGLO*GDP	0.266***	0.045	3.261	(0.008)
lnPGLO*GDP	0.426***	0.033	2.054	(0.000)
lnK	0.314***	0.051	3.869	(0.005)
lnL	-0.156***	0.083	-5.085	(0.000)
ECM(-1)	-0.212***	0.0257	-47.128	(-0.009)

**Note:** ***, ** and * indicate statistical significance at 1% level, 5% level and 10% level respectively, where inside in the parentheses are probability values.

The results also point out that decentralized globalization (economic, social, and political globalization) has significantly boosted renewable energy consumption in emerging Asian economies. These globalization practices thus play an important role in renewable energy consumption in emerging Asian economies. For every 1 percentage point increase in economic, social and political globalization, renewable energy consumption will increase significantly by 0.488 percentage points, 0.383 percentage points and 0.373 percentage points, respectively. This result is consistent with [88, 89]. The results show that economic globalization increases the consumption of renewable energy by promoting the import of advanced and friendly technologies. Evidence for the strong impact of social globalization factors on renewable energy consumption is based on the fact that globalized social norms have increased the dependence of emerging Asian countries on renewable energy consumption. In terms of political globalization, emerging economies in Asia have recently highlighted renewable energy plans, and politicians have shown interest in shifting their reliance on renewable energy.

However, the nonlinear effect model reflects that the main term of economic, social and political globalization has a significant negative impact on renewable energy consumption, while its square term has a significant incremental impact on renewable energy consumption. This result suggests a U-shaped relationship between globalization indicators and renewable energy consumption. Thus, renewable energy decreases at the beginning of globalization, but renewable energy consumption increases after globalization reaches a certain threshold. The interaction of political, economic, and social globalization with economic growth has also witnessed an increase in renewable energy consumption, which supports the scale effect hypothesis.

The AMG estimator is used to check the robustness of the long-term results of renewable energy models through CS-ARDL tests. Table 11 highlights the AMG estimation results, reflecting broad agreement with the CS-ARDL results in terms of coefficient signs.

**Table 11:** Long-term AMG estimation results for robustness checks.

Variables	Coefficients	Standard error	Z-value	P-value
lnRE = f(InGDP, InSGLO, InEGLO, InPGLO, lnK, lnL)				
lnGDP	0.157***	0.029	4.014	(0.005)
lnSGLO	0.305***	0.061	5.062	(0.004)
lnEGLO	0.328***	0.037	4.244	(0.001)
lnPGLO	0.241***	0.054	3.091	(0.000)
lnK	0.266***	0.081	2.071	(0.008)
lnL	-0.469***	0.032	-5.095	(0.000)
Constant	-4.218***	0.063	-3.352	(0.005)
Wald	51.073***			
RMSE (sigma)	0.031			
InRE = f(InGDP, InSGLO, lnEGLO, InPGLO, lnSGLO^2^, lnEGLO^2^, lnPGLO^2^, lnK, lnL)				
lnGDP	0.352***	0.041	4.136	(0.007)
lnSGLO	-0.131**	0.081	-4.012	(-0.021)
lnEGLO	-0.291***	0.041	-5.195	(-0.003)
lnPGLO	-0.296***	0.042	3.082	(0.004)
lnSGLO^2^	0.687***	0.083	4.585	(0.000)
lnEGLO^2^	0.516***	0.068	3.728	(0.000)
lnPGLO^2^	0.715**	0.059	4.074	(0.042)
lnK	0.516***	0.042	3.691	(0.005)
lnL	-0.317***	0.041	-3.087	(0.000)
Constant	-0.526***	0.057	4.068	(0.009)
Wald	93.074***			
RMSE (sigma)	0.061			
InRE = f(InGDP, InSGLO, lnEGLO, InPGLO, lnSGLO*lnGDP, lnEGLO*lnGDP, lnPGLO*lnGDP, lnK, lnL)				
lnGDP	0.132***	0.074	3.173	(0.007)
lnSGLO	0.371**	0.081	3.157	(0.032)
lnEGLO	0.124***	0.030	5.086	(0.000)
lnPGLO	0.416***	0.063	4.027	(0.003)
lnSGLO*GDP	0.457***	0.073	4.076	(0.006)
lnEGLO*GDP	0.117**	0.062	3.177	(0.048)
lnPGLO*GDP	0.426***	0.053	3.648	(0.000)
lnK	0.174***	0.031	4.048	(0.009)
lnL	-0.286***	0.078	-5.249	(0.000)
Constant	-0.182***	0.048	-4.514	(0.008)
Wald	73.41***			
RMSE (sigma)	0.031			

**Note:** ***, ** and * indicate statistical significance at 1% level, 5% level and 10% level respectively, where inside in the parentheses are probability values.

Next, the Dumitrescu-Hurlin causality approach was used to detect causality among our variables of interest for specific emerging Asian economies, and the results are highlighted in Table 12. Renewable energy and economic growth have bidirectional causality, thus supporting the feedback hypothesis. There are also two-way causal relationships between social globalization and economic growth, and between economic growth and economic globalization. Moreover, there is a one-way causal relationship from renewable energy to political globalization, from social globalization to capital formation, from economic globalization to renewable energy consumption and capital formation. There are also one-way causal relationships from political globalization to economic growth, from capital accumulation to economic growth, renewable energy consumption, and social globalization.

**Table 12:** Dumitrescu-Hurlin panel causality test results.

Variables	lnGDP	lnRE	lnSGLO	lnEGLO	lnPGLO	lnK	lnL
InGDP	--------	1.078*** (0.002)	2.713** (0.032)	2.055*** (0.005)	3.732 (0.123)	1.071 (0.481)	2.179 (0.265)
InRE	2.081** (0.034)	--------	2.161 (0.284)	2.291 (0.375)	1.273*** (0.000)	3.327 (0.413)	1.279 (0.217)
InSGLO	3.071*** (0.001)	1.465** (0.032)	---------	1.785 (0.364)	2.107 (0.274)	2.328*** (0.000)	1.278 (0.325)
lnEGLO	1.097** (0.042)	1.167*** (0.000)	2.161 (0.535)	-----------	2.162 (0.265)	3.185** (0.046)	2.167 (0.214)
InPGLO	3.071*** (0.007)	3.084 (0.277)	2.185 (0.384)	2.978 (0.371)	----------	3.095 (0.174)	2.890 (0.217)
lnK	4.523*** (0.000)	3.276** (0.036)	1.620*** (0.000)	3.544 (0.485)	3.224 (0.544)	-----------	0.315 (0.421)
lnL	2.178 (0.215)	4.156 (0.316)	2.167 (0.217)	1.365 (0.214)	4.135 (0.314)	2.176 (0.216)	-----------

**Note:** ***, ** and * indicate statistical significance at 1% level, 5% level and 10% level respectively, where inside in the parentheses are probability values.

## 5. Conclusion and policy implications

Using the CS-ARDL approach, this study examines the impact of globalization indicators on the link between renewable energy consumption and economic growth in six emerging Asian economies over the period 1975 to 2020. The research analysis draws several findings. First, the results of the economic growth model show that renewable energy consumption has a significant contribution to economic growth. The conclusions further point out that economic and political globalization firmly hold back economic growth, while social globalization directly promotes economic growth in selected Asian emerging economies. The non-linear impact of political, economic and social globalization on economic growth shows that political and economic globalization significantly promotes economic growth, while social globalization significantly reduces economic growth. However, the square of political and economic globalization significantly reduces economic growth, while the square of social globalization significantly boosts economic growth in emerging Asian economies. This result clearly proves the validity of the inverted U-shaped relationship between political globalization, economic globalization and economic growth, and the legitimacy of the U-shaped relationship between social globalization and economic growth. The study also found that economic, social and political globalization moderated the impact of renewable energy on boosting economic growth.

Second, for the renewable energy consumption model, it is revealed that economic growth significantly promotes renewable energy consumption. The results also point out that decentralized globalization (economic, social, and political globalization) has significantly boosted renewable energy consumption in emerging Asian economies. However, the nonlinear effect model reflects that the main term of economic, social and political globalization has a significant negative impact on renewable energy consumption, while its square term has a significant incremental impact on renewable energy consumption. This result suggests a U-shaped relationship between globalization indicators and renewable energy consumption. The interaction of political, economic, and social globalization with economic growth has also witnessed an increase in renewable energy consumption, which supports the scale effect hypothesis. The causality test concludes that there is a two-way causal relationship between renewable energy consumption and economic growth, thus supporting the feedback hypothesis.

The findings provide important policy implications for Asian emerging economies. Existing evidence in this study suggests that economic and political globalization promotes short-term economic growth but hurts long-term economic growth. However, social globalization inhibits economic growth in the short run and promotes economic growth in the long run. Although globalization brings short-term economic benefits, it is crucial for policymakers to implement favorable policies to limit the adverse effects of economic globalization on long-term economic growth. Economic globalization drives long-term economic growth in emerging Asian economies, which is critical for policymakers to formulate corporate policies that encourage a deeper understanding of economic sectors with dynamic comparative advantages in terms of output growth. Furthermore, given the technological impact of globalization, ensuring the transfer of technological innovation to less technologically innovative productive sectors is imperative to foster long-term economic growth. Finally, economic globalization in light of income inequality and unemployment may hinder long-term economic growth. Policymakers have an obligation to use necessary social interventions as a tool to provide a "safety net" for those harmed by economic globalization. Building on existing politically and economically extractive institutions remains crucial for globalization to foster long-term economic growth in emerging Asia. Renewable energy consumption interacts with economic, social, and political globalization to boost economic growth in emerging Asian economies. This means that productivity and commodity flow in the economic globalization based on advanced and friendly technology, will not only promote economic growth, but also bring about sustainable development of the environment.

The nonlinear effect model of renewable energy consumption reflects a U-shaped relationship between globalization indicators and renewable energy consumption. Thus, globalization indicators only worsen renewable energy efficiency in the short run, while improving renewable energy efficiency in the long run. Thus, from a policy perspective, it has been recommended that policymakers in the Asian emerging economies should not misjudge the effects of globalization in renewable energy demand models while formulating and implementing environmental conservation policies.

For future research directions, the role of renewable energy consumption in the link between fragmented globalization and environmental sustainability should be explored for Asian emerging economies. In addition, an N-shaped EKC assumption between globalization indicators and renewable energy consumption should be established for the specific panel to predict future environmental protection measures.
